# The Comprehensive Analysis of Hub Gene ARRB2 in Prostate Cancer

**DOI:** 10.1155/2022/8518378

**Published:** 2022-10-15

**Authors:** Bing Zhou, Hong Song, Wuqin Xu, Yanbin Zhang, Yinhua Liu, Wei Qi

**Affiliations:** ^1^Department of Pathology, Yijishan Hospital, The First Affiliated Hospital of Wannan Medical College, Wuhu, Anhui 241001, China; ^2^Department of Urology, Hefei Hospital Affiliated to Anhui Medical University (The Second People's Hospital of Hefei), Hefei, Anhui Province 230011, China

## Abstract

**Methods:**

The differential expressed genes (DEGs) were screened from the gene expression profile GSE30994 related to PRAD and then analyzed by protein-protein interaction (PPI) to screen the hub gene. Subsequently, the relation between hub gene and pan cancers, PRAD prognosis, and immunotherapy was analyzed. Besides, the effects of hub gene on the growth and metastasis of PRAD cell lines and inflammatory factors (IFs) were detected by functional experiments.

**Results:**

276 upregulated and 1,861 downregulated DEGs were analyzed from GSE30994 gene expression profiles. Through enrichment analysis, it was found that upregulated DEGs were significantly enriched in nitric oxide-mediated signal transduction, insulin signaling pathway, etc. Through PPI networks, ARRB2 was determined as the hub gene that was highly expressed in pan cancers, including PRAD, and contributed to poor prognosis of PRAD patients. Immunoassay showed that ARRB2 was associated with B cells, NK cells, endothelial cells, etc. and also connected with tumor-infiltrating lymphocytes (TILs). Next, the signature model analysis revealed that ARRB2 had a clinical value in predicting PRAD prognosis. In functional experiments, ARRB2 was highly expressed in PRAD cell lines, promoted PRAD cell growth and metastasis, and positively associated with IFs.

**Conclusion:**

ARRB2 has a good prognostic ability in PRAD, and it could be a potential target of PRAD immunotherapy, which offers new directions for PRAD research.

## 1. Background

As the most frequent malignant tumor in the male genitourinary system, prostate adenocarcinoma (PRAD) results from the malignant proliferation of prostate epithelial cells [1]. PRAD usually occurs in elderly males with family heredity, often manifested as abnormal urination, pelvic discomfort, erectile dysfunction, and so on [2]. Advanced PRAD metastasis can happen in the bone, causing bone pain or pathological fracture or paraplegia, and even invading the bone marrow [3]. Clinically, it is divided into ductal adenocarcinoma, actinoid adenocarcinoma, squamous cell carcinoma, urothelial carcinoma, and adenosquamous carcinoma according to its pathological type [4]. For patients with early localized PRAD, they can get radical treatment through surgery or radiotherapy to achieve a good prognosis, and the 5-year survival rate can reach over 90% [3, 5]. However, for patients with advanced metastatic PRAD, it is still very difficult to have a good prognosis. We performed a literature search using PubMed and Embase while referencing EAU guidelines for the management of Peyronie's disease for studies published 1980-2020 [6, 7].

Many previous studies have shown that the occurrence and progression of PRAD are related to mutated genes and their abnormal expressions [8, 9]. Zu-Cheng et al. studied the clinical application of miR-1 in PRAD and related molecular mechanisms [10]. Altwaijry et al. proposed in the study that TP53 and GSTP1 were involved in gene mutations, thereby promoting the development of PRAD [11]. Recent studies have indicated that BRCA germline mutations in PRAD are particularly important in the clinical setting, primarily because carriers have an increased risk of developing PRAD compared with noncarriers, and PRAD with BRCA-associated mutations characterized by the clinical prognosis is worse [9]. Clinically, PRAD patients are screened by magnetic resonance, functional imaging technology, prostate-specific antigen, biomarkers, and other methods and then treated by immunotherapy, knockout of male hormones, chemotherapy, and others [12–14]. Specific and sensitive biomarkers can not only quickly and accurately facilitate the diagnosis and treatment of patients [15, 16] but is also very useful for a comprehensive understanding of molecular pathogenesis [17]. However, despite the increasingly advanced medical technology in PRAD, effective biomarkers for clinical diagnosis, treatment, and prognosis are still lacking.

High-throughput gene microarray technology is usually used to study molecular biology, which is of great significance to the field of genomics. This technology is widely used to find candidate genes for diseases and provide a more convenient method for the diagnosis and monitor tumor diseases [18]. In the present study, to identify specific and sensitive molecular biomarkers in PRAD pathogenesis, we first identified differentially expressed genes (DEGs) in the GSE30994 gene expression profile. On this basis, the functional enrichment analyses on DEGs were performed to identify the hub gene. Then, the hub gene was proved to be a promising biomarker for PRAD immunotherapy and prognosis by bioinformatics analysis and experiments.

## 2. Material and Methods

### 2.1. Microarray Data Acquisition and Identification of DEGs

From the Gene Expressed Omnibus (GEO) database, the GSE30994 gene expression file was downloaded, containing 3 sets of normal prostate biopsy and 3 sets of PRAD biopsy. By GEO2R, we analyzed these samples. DEGs were screened according to the criteria of log_2_FC > 1 (upregulation) and log_2_FC < −1 (downregulation). The *P* value <0.05 indicated statistical significance. After that, ImageGP was used to generate the volcano and heat maps of these DEGs.

### 2.2. Functional Enrichment Analysis of DEGs

Gene Ontology (GO) annotation and Kyoto Encyclopedia of Genes and Genomes (KEGG) pathway are common functional enrichment analyses for DEGs. The former mainly provides annotations for GO terms, including biological process (BP), cell component (CC), and molecular function (MF). The latter helps to further decipher the function of genes. Based on this, we performed GO and KEGG pathway enrichment analysis on the screened upregulated DEGs by the DAVID database to determine their biological functions. The results of downregulated DEGs were not displayed due to their nonsignificance.

### 2.3. PPI Network Analysis

As an online tool, the search tool for retrieving interacting genes (STRING) [19] is used to evaluate the integrated PPI information. The interactive relationships among upregulated DEGs were evaluated, and the hub gene was identified according to the degree values. At last, ARRB2 was determined as the hub gene related to PRAD.

### 2.4. Expression Verification of the ARRB2 Gene in Pan Cancers

The Genotype-Tissue Expression (GTEx) database is often used in conjunction with the Cancer Genome Atlas (TCGA) database for single-gene expression analysis in pan cancers. This time, the levels of ARRB2 in various normal and tumor tissues were analyzed by TCGA and GTEx databases. Subsequently, PRAD samples were downloaded from the TCGA database, and the expression differences of ARRB2 in different clinical parameters (sample types, metastasis status, TP53 mutation status) in PRAD were compared.

### 2.5. Kaplan-Meier (KM) Plotter Analysis of ARRB2 in PRAD

To test the prognostic level of the ARRB2 gene, we performed a Cox analysis of the ARRB2 gene in pan cancers and calculated the corresponding *P* value and hazard ratio (HR) with a 90% confidence interval (CI). The results obtained were statistically significant when *P* < 0.05. Next, 246 PRAD samples with high ARRB2 expression and 246 PRAD samples with low ARRB2 expression were downloaded from the TCGA database, and the effects of differently expressed ARRB2 on the overall survival (OS) and disease-free survival (DFS) of PARD patients were analyzed by KM plotter.

### 2.6. Immunoassay on ARRB2 in PRAD

As a comprehensive resource, Tumor Immune Estimation Resource (TIMER) webserver was used for systematically analyzing the immune infiltration of different cancer types, which was convenient for grasping the immunological, clinical, and genomic characteristics of tumors. Herein, we first used the “immunedeconv” package of the *R* software, to analyze the infiltration levels of 6 immune cells in the high- and low-ARRB2-expressing groups. The correlation between ARRB2 and immune cells was then evaluated according to Spearman's correlation analysis. Subsequently, on the Tumor and Immune System Interaction Database (TISIDB) website, we successively analyzed the correlation between ARRB2 and tumor-infiltrating lymphocytes (TILs), immunosuppressants, immunostimulants, chemokines, and receptors. Besides, the relation between TILs (Treg, Tfh, Tcm CD4, and Tem CD8) and PRAD was explored by Spearman's correlation analysis. Finally, the levels of immune checkpoint molecules (CD274, HAVCR2, CTLA4, LAG3, PDCD1LG2, PDCD1, TIGIT, SIGLEC15) in different ARRB2 expression groups were examined by Wilcoxon.

### 2.7. Establishment of ARRB2 Prognostic Signature Model

Significant clinical prognostic factors of PRAD were analyzed by univariate and multivariate Cox regression, and the corresponding *P* value of each variable was displayed by forest plots. Based on this result, a nomogram was built using the “rms” package to predict 1-, 3-, and 5-year survival conditions of PRAD patients, and a concordance index (*C*-index) was calculated. A calibration curve was mapped to observe the predictive accuracy of the nomogram. Next, PRAD patient samples were divided into high-risk and low-risk groups according to ARRB2 expressions, namely, 248 ARRB2 high-expression and 248 low-expression samples, the effect of different expression groups on the progression-free survival (PFS) rate of patients was evaluated by KM survival analysis, and the relevant hazard ratio (HR) and the median time of the two groups were calculated. Then, the receiver operating characteristic (ROC) curve was constructed by the “survivalROC” package of the *R* software to calculate the area under curve (AUC) values of the patients at 1, 3, and 5 years to evaluate the prognostic prediction efficiency.

## 3. Cell Lines and Cell Culture

Human PRAD cell lines (LNCap, DU145, and PC-3) and pertinent normal cells (RWPE-1) were from Fenghui Biotechnology Co., Ltd. (Hunan, China). They were cultivated in DMEM (Gibco, USA) with 10% FBS (HyClone, USA) at 37°C.

### 3.1. Cell Transfection

Lipofectamine 2000 (Invitrogen) was used for cell transfection. ARRB2 in PRAD cells was transfected by siRNAs (si-ARRB2 #1, si-ARRB2 #2 and si-ARRB2 #3) and overexpression vector (over-ARRB2), respectively, as instructed.

### 3.2. Quantitative Real-Time PCR (qRT-PCR)

qRT-PCR was conducted by SYBR Premix Extaq (Takara, USA). The endogenous *β*-actin expression was used as a standardized control. The 2^-*ΔΔ*Ct^ method was adopted to calculate the pertinent expression.

### 3.3. CCK-8 (Cell Count Kit-8) Test

Cells were seeded into 96-well plates with 1 × 10^3^ cells per well. CCK-8 was added in an incubator at 37°C and 5% CO_2_ in the dark. The optical density (OD) was measured by a 450 nm microplate analyzer at 1, 2, 3, and 4 days, respectively.

### 3.4. Transwell Assay

For migration assay, cells were seeded into the upper chamber containing DMEM and 10% FBS and the lower chamber with about 600 *μ*L DMEM containing 10% FBS in a CO_2_ incubator at 37°C for 24 h. After that, the upper was removed and carefully wiped off from the membrane with a cotton swab. The cells were washed twice in preheated PBS solution at 37°C and fixed with 4% paraformaldehyde for 30 min. Then, they were dyed with hematoxylin for 5 minutes. For the invasion assay, the steps were the same as the above, except for the precoated 50 *μ*l of Matrigel in the upper chamber membranes. The cells were observed under a microscope.

### 3.5. Statistical Analysis

All data were determined as the mean standard deviation in this study, and statistical comparisons between groups were made using one-way ANOVA and Student's *t*-test.

Statistical analyses were performed with GraphPad Prism 6.0 software, and data were expressed as mean ± SD. Statistical comparisons were made by one-way analysis of variance (ANOVA), and *P* < 0.05 instructed a statistically significant difference.

## 4. Results

### 4.1. Identification of DEGs

There were 3 normal prostate biopsies and 3 PRAD biopsies in this study. We obtained 2,137 DEGs by making use of the GEO2R online analysis tool, of which 276 were up and 1,861 were down (Figure 1(a)).  Figure 1(b) shows the expressions of these DEGs in 6 samples.

### 4.2. GO Function and KEGG Pathway Enrichment Analysis

To a deeper understanding of the upregulated DEGs, we applied DAVID to perform the GO and KEGG pathway enrichment analyses. In BP, these genes were mainly enriched in arginine metabolic process, nitric oxide-mediated signal transduction, regulation of heart contraction, protein ADP-ribosylation, regulation of cardiac conduction, and lipoxin biosynthetic process (Figure 1(c)). In CC, these genes were significantly enriched in the neurotransmitter receptor complex, U2-type prespliceosome, platelet dense granule, spliceosomal snRNP complex, etc. (Figure 1(d)). In MF, these genes were significantly abundant in arginine binding, NADPH-hemoprotein reductase activity, etc. (Figure 1(e)). According to the bubble chart of the KEGG enrichment pathway in Figure 1(f), it was obvious that these upregulated DEGs were significantly abundant in the sphingolipid, apelin, insulin, and HIF-1 signaling pathways.

### 4.3. Hub Gene Identification from the PPI Network

Based on the public database, we used STRING to establish a PPI network of significantly upregulated genes (Figure 1(g)). This PPI network included 237 nodes and 159 edges, of which ARRB2 had the highest degree of 9; so, ARRB2 was the hub gene in this study.

### 4.4. Expression Analysis of ARRB2 in Pan Cancers and PRAD Samples with Different Factors

As shown in Figure 2(a), it could be seen from the results of the box plot that the levels of ARRB2 in many tumor tissues were significantly higher than those in normal tissues, including PRAD, which confirmed that ARRB2 was widely involved in the development of tumors. Next, the results in Figure 2(b) showed that ARRB2 was highly expressed in PRAD primary tumors. Furthermore, ARRB2 was highly expressed in N1 and TP53-nonmutant groups compared with N0 and TP53-mutant, suggesting that the level of this gene increased with tumor progression (Figures 2(c) and 2(d)).

### 4.5. KM Analysis on ARRB2 in PRAD Prognosis

According to the results of Cox regression analysis, we found that ARRB2 was significantly different in lung adenocarcinoma (LUAD, *P* = 0.0260), pancreatic cancer (PAAD, *P* = 0.0155), and PRAD (*P* = 0.0003). After that, it was found that the OS and DFS rates of ARRB2 patients in the high expression group were poor; so, we supposed that the high expression of ARRB2 was connected with the poor survival rate of PRAD patients (Figures 3(b) and 3(c)).

### 4.6. ARRB2 Was Associated with the Immune Infiltration in PRAD

According to the results of the immunoassay, we found that the expressions of ARRB2 in B cell, neutrophil, T cell CD4+, myeloid dendritic cell, and macrophage were significantly different. Moreover, the TIMER score values of immune cells in the ARRB2 high expression group were generally higher (Figure 4(a)). Spearman correlation analysis indicated that ARRB2 expressions were positively correlated with the expressions of B cell (*ρ*_Spearman_ = 0.12), NK cell (*ρ*_Spearman_ = 0.16), endothelial cell (*ρ*_Spearman_ = 0.35), and macrophage (*ρ*_Spearman_ = 0.65), while negatively correlated with uncharacterized cell (*ρ*_Spearman_ = −0.28, Figure 4(b)). Subsequently, based on the heat map of the correlation analysis between TILs and PRAD (Figure 4(c)), we performed the correlation analysis between ARRB2 and the 4 cells, Treg, Tfh, Tcm CD4, and Tem CD8. The results in Figures 4(d)–4(g) displayed that Tfh (rho = 0.445) had the highest correlation with ARRB2, followed by Tem CD8 (rho = 0.42), Tcm CD4 (rho = 0.373), and Treg (rho = 0.362). Among the immunosuppressants, we found that ARRB2 had the strongest correlation with ADORA2A, HAVCR2, and LGALSP (Figure 5(a)). Similarly, in immunostimulants, it was observed that ARRB2 in PARD was positively correlated with C10orf54, CD27, etc. and negatively correlated with NT5E, PVR, etc. (Figure 5(b)). Among chemokines, we found that the ARRB2 gene was significantly correlated with HLA-DMA and HLA-DPB1 (Figure 5(c)). In receptor analysis, significant correlations were observed between ARRB2 and CCR5, CCR7, and CCR10 (Figure 5(d)). Finally, according to Figure 5(e), it could be found that in the results of immune checkpoint research, ARRB2 with high expression levels had a significantly positive relation with CD274, HAVCR2, CTLA4, LAG3, TIGIT, PDCD1, and PDCD1LG2, except SIGLEC15. Taken together, we could determine that ARRB2 was associated with immune infiltration in PRAD.

### 4.7. The Establishment of PRAD Prognostic Signature Model with ARRB2

The forest plots in Figures 6(a) and 6(b) assessed the prognostic impact of ARRB2 and different clinical variables on PRAD patients. According to the *P* < 0.05 criterion, ARRB2 (*P* = 0.00471) and pT stage (*P* = 0.00002) were obtained as key factors. Then, based on these two variables, we constructed a nomogram through the “rms” package to detect the effect of key variables on the 1-, 3-, and 5-year survival time for PRAD patients and obtained a *C*-index of 0.689 (Figure 6(c)). Moreover, the calibration curve of the nomogram also showed that the 1-, 3-, and 5-year survival of PRAD patients was close to the calibration curve (Figure 6(d)). Subsequently, we divided the PRAD patient samples into the ARRB2 high group and low group (Figure 6(e)) and found that the PRAD patients in the ARRB2 high group had a poorer prognosis, with a median time of 5.8 years and an HR of 2.206 (>1), indicating that ARRB2 was a risk factor for PRAD prognosis (Figure 6(f)). Finally, the results of the ROC curve showed that the AUC value corresponding to the 5-year survival of PRAD patients was the highest, which was 0.711 (Figure 6(g)). In conclusion, the analysis of the prognostic signature model showed that ARRB2 had a certain predictive ability for the prognosis of PRAD patients.

### 4.8. Upregulation of ARRB2 in PRAD Cell Lines

Based on the detection of ARRB2 levels in TIMER, we carried out qRT-PRADR assays to measure its expressions in PRAD cell lines (DU145, LNCap, and PC-3) and normal prostate cells (RWPE-1). As Figure 7(a) indicated, ARRB2 was significantly upregulated in PRAD cells than in normal prostate cells, particularly in DU145 and PC-3, which conformed to the results in TIMER.

### 4.9. Effects of ARRB2 Expression on the Proliferation, Migration, and Invasion of PRAD Cells

Next, we applied functional experiments to further study the effects of ARRB2 in PRAD. First, si-ARRB2 #1, si-ARRB2 #2, and si-ARRB2 #3 were transfected into DU145 and PC-3 to silence the ARRB2 expression, and then ARRB2 was overexpressed by over-ARRB2 in DU145 cells (Figures 7(b) and 7(e)). Si-ARRB2 #1 was chosen for its great knockdown efficiency. After this, CCK-8 showed that si-ARRB2 #1 could slow down the proliferation rate of PRAD cells (Figures 7(c) and 7(d)), while overexpressed ARRB2 promoted cell proliferation (Figure 7(f)). Besides, transwell assays demonstrated that si-ARRB2 #1 could also abate PRAD cell invasion and migration (Figures 8(a) and 8(b)), whereas overexpressed ARRB2 had a promoting effect on PRAD cell migration and invasion (Figure 8(c)). These results conveyed that ARRB2 might be involved in the oncogenic process of PRAD.

### 4.10. ARRB2 in PRAD Cells Positively Regulated IFs

Next, we measured the levels of IFs (IL-6 and TNF-*α*) in PRAD cell lines by qRT-PCR and found that these two IFs were both highly expressed in PRAD (Figures 9(a) and 9(b)). Moreover, the results of Figures 9(c)–9(f) showed that the expression levels of IL-6 and TNF-*α* in DU145 cells were positively correlated with the expression of ARRB2, indicating that ARRB2 had a positive regulatory effect on IFs.

## 5. Discussion

As one of the malignant tumors that often occur in middle-aged and elderly men, PRAD has an increasing trend of morbidity and mortality in recent years [20]. Although medical technology advances have improved the treatment of PRAD, the overall prognosis is still unsatisfying [21]. Therefore, the study on the specific and sensitive PRAD biomarkers and new therapies needs to be carried out. Herein, we applied high-throughput sequencing to this research to better understand the pathogenesis of PRAD and search for specific biomarkers and new therapies. Through the analysis on the GSE30994 database, we obtained 2,173 DEGs in total, of which 276 were upregulated and 1,861 were downregulated. For the significance of results, the upregulated DEGs were adopted for further research.

According to the enrichment results of GO term and KEGG pathway on upregulated DEGs, it was demonstrated that these genes were significantly enriched in BP in nitric oxide-mediated signal transduction [22], arginine metabolic process, regulation of cardiac conduction, negative regulation of calcium-mediated signaling, etc. In the KEGG pathway, we identified that these genes were significantly enriched in four pathways, apelin [23], sphinolipid, insulin [24], and HIF-1 [25]. Among them, the study by Nandeesha et al. pointed out that factors, such as hormone imbalance, obesity, and family genetic history, were risk factors for the onset of PRAD and verified the relationship between insulin and PRAD [26]. The results showed that the growth factor pathway, signal transduction mechanism, and dyslipidemia of insulin were related to the pathogenesis of PRAD. Many other studies have mentioned that interference with insulin-like growth factor signaling can be used as one of the PRAD treatments, which also confirms the mechanism of the insulin signaling pathway in PRAD from the side [27]. Not only that, Pan and Chen analyzed the relationship between HIF-1 and PRAD, and concluded that HIF-1 not only participated in the biological processes of PRAD [28], such as angiogenesis, cell proliferation, and glucose metabolism, but also in P53, P21, and signal transduction pathway. Therefore, the insulin signaling pathway and HIF-1 signaling pathway might be the predictors in the diagnosis and treatment of PRAD, providing new directions for clinical patients.

In the present study, we identified ARRB2 as a major target gene through the PPI network. ARRB2, whose full name is arrestin beta 2, is also known as ARB2, ARR2, or BARR2, usually associated with diseases like WHIM syndrome and cryptococcal meningitis [29]. The study by Kallifatidis et al. verifies that ARRB2 is involved in leukemia and medulloblastoma and combines with other molecular compounds [30], indicating that it can regulate the characteristics of stem cells and might be used as a potential target in tumor treatment. In our study, the expressions of ARRB2 in various tumors were obviously higher than that in normal tissues, ARRB2 was highly expressed in PRAD tumor tissues, and its expression was significantly different in different nodal metastasis and TP53 mutation status. KM curve demonstrated that patients with the low ARRB2 expression had better OS and DFS. Moreover, we applied ARRB2 and PRAD clinical factors to construct a nomogram to predict 1-, 3-, and 5-year survival status. The results showed that this nomogram had a good predictive ability. Based on the above findings, we concluded that ARRB2 was an oncogene in PRAD progression, and it could be a prognostic biomarker for PRAD patients. This speculation was proved in the experiments, in which si-ARRB2 could inhibit the cell growth, invasion, and migration, while over-ARRB2 could promote them.

With the rapid development of tumor immunology, a large number of studies on the interaction between tumor genes and immunity have become a research hotspot. For example, Hu et al. performed an immunological and prognostic analysis of the YTHDF1 gene in cancer based on a public dataset repository and found a significant association between the expression of YTHDF1 and TILs, and the coexpression network of YHDF1 was also involved in the regulation of immune responses [31]. The study of Huang et al. confirmed 5 chemokines related to the occurrence, progression, prognosis, and immune infiltration of cutaneous melanoma, namely, CXCL9, CXCL10, CXCL13, CCL4, and CCL5 [32]. In addition, other studies have confirmed that the expression of AQP3 was significantly associated with TILs in LUAD, inferring that this gene could be used as a prognostic and survival biomarker in LUAD patients [33]. Based on this, it is feasible to study the effect of ARRB2 on PRAD development from the perspective of immune analysis. Through the TIMER database, we found that the expression of ARRB2 was significantly different in B cells, T cell CD4+, neutrophils, macrophages, and myeloid dendritic cells. In addition, we found that the immune infiltration level of ARRB2 was associated with many immune factors. In the immune checkpoint analysis, ARRB2 with different expression levels was found to be significantly different in CD274, HAVCR2, and so on. Therefore, we infer that the expression of ARRB2 affects the immune cells in PRAD, and it has the potential to be one of the targets of PRAD immunotherapy.

Several studies have suggested that IFs are related to the development and prognosis of cancer, among which TNF-*α* and IL-6 are the most typical cytokines related to inflammation, which can play an important role in host defense by regulating immune and inflammatory responses [34, 35]. For example, the study by Garrido et al. demonstrated IL-6 and TNF-*α* were highly expressed in high-risk PRAD samples [36]. Zhou et al. found that the expression levels of TNF-*α* and IL-6 could affect the change in Gleason score (GS) of PRAD. TNF-*α* had a positive correlation with GS upgrading, and IL-6 had a negative correlation with GS upgrading [37]. In our cell experiments, TNF-*α* and IL-6 were highly expressed in PRAD cell lines and positively regulated by ARRB2, suggesting that ARRB2 could affect PRAD tumor progression by regulating the expression of IFs.

In summary, we identified a total of 276 upregulated DEGs and 1861 downregulated DEGs, and ARRB2 was further chosen as the target gene by the PPI network. Through bioinformatics analysis, ARRB2 is proved to be an oncogene in PRAD development, and it could be a potential target of PRAD immunotherapy and biomarker for the prognosis of PRAD patients. However, this study has certain limitations and lacks further validation in vivo experiments. In the follow-up study, we plan to validate our findings in sufficient clinical samples and animal experiments. In addition, it is necessary to further elucidate the role of ARRB2 in PRAD. Mechanism. Through follow-up in-depth research, we hope that our findings can play a role in the diagnosis and elucidation of the pathogenesis of PRAD.

## Figures and Tables

**Figure 1:** Screening and analysis of DEGs in the GSE30994 dataset. (a) Volcano map. (b) Heat map. The upregulated DEGs and downregulated DEGs in 6 sample data. (c)–(e) GO term enrichment analysis on upregulated DEGs in BP, CC, and MF, respectively. (f) The top 10 pathways of upregulated DEGs enriched in KEGG. (g) PPI network of upregulated DEGs. The red node was the key gene-ARRB2.

**Figure 2:** Expression validation of ARRB2 in pan cancers. (a) The expression levels of ARRB2 in normal tissues and tumor tissues, ns: not significant. (b)–(d) Expression level analysis of ARRB2 in sample types, nodal metastasis status, and TP53 mutation status in PARD. ^∗^*P* < 0.05, ^∗∗^*P* < 0.01, ^∗∗∗^*P* < 0.001.

**Figure 3:** The prognostic value of ARRB2 in PRAD. (a) Cox analysis of ARRB2 in pan cancers. (b) Correlation analysis of ARRB2 expression level and OS in PRAD patients. (c) Correlation analysis of ARRB2 expression level and DFS in PRAD patients.

**Figure 4:** The relationship between ARRB2 expression and PRAD immune infiltration level. (a) Immune cell infiltration levels in high and low ARRB2 expression groups by the TIMER database. (b) Spearman correlation analysis of ARRB2 and immune cells. The abscissa represents the expression score distribution of genes, the ordinate represents the immune score distribution, and *ρ*_Spearman_ is the correlation coefficient. (c) Correlation between ARRB2 and immune infiltration levels. (d)–(g) Spearman analysis of the relationship between ARRB2 and Treg, Tfh, Tcm CD4, and Tem CD8.

**Figure 5:** Correlation analysis between ARRB2 expression and immune markers in PRAD. (a)–(d) Heat maps show the correlation of ARRB2 with immunosuppressants, immunostimulants, chemokines, and receptors, respectively. (e) Boxplot. Expression distribution of immune checkpoint genes in the high ARRB2 expression group and low ARRB2 expression group. ^∗∗∗^*P* < 0.001.

**Figure 6:** The establishment of the prognostic signature model. (a, b) Forest plots for univariate and multivariate Cox analyses, respectively. (c) Nomogram of the effect of key clinical variables on PRAD patient survival time. (d) Calibration curves for the nomogram predicting 1-, 3-, and 5-year survival. (e) Scatter plot of risk analysis, with red for high-risk groups and blue for low-risk groups. (f) KM survival curve graph of high ARRB2 and low ARRB2. The median time was 5.8. (g) ROC curve analysis. AUC values under different color curves represent the prognostic prediction ability of different survival times.

**Figure 7:** The effect of ARRB2 on PRAD cell proliferation. (a) ARRB2 mRNA expressions in normal prostate cells and PRAD cells. (b) Knockdown of the ARRB2 expression in DU145 and PC-3 cell lines by si-ARRB2 #1, si-ARRB2 #2, and si-ARRB2 #3. (c, d) The effect of si-ARRB2 #1 on the proliferation of DU145 cells was examined. (e) ARRB2 was overexpressed in the DU145 cell line. (f) The effect of the ARRB2 overexpression on the proliferation of DU145 cells. ^∗^*P* < 0.05, ^∗∗^*P* < 0.01.

**Figure 8:** The effect of ARRB2 on PRAD cell migration and invasion. (a) Si-ARRB2 #1 knocked down the DU145 cell invasion and migration. (b) Si-ARRB2 #1 knocked down the PC-3 cell invasion and migration. (c) Over-ARRB2 #1 promoted the DU145 cell invasion and migration. ^∗^*P* < 0.05.

**Figure 9:** ARRB2 could promote the expression levels of IFs in PRAD. (a, b) Expression levels of IL 6 and TNF-*α* in PRAD cell lines. (c, d) The knockdown regulation of IL 6 and TNF-*α* in PRAD cells by si-ARRB2 #1. (e, f) The upregulation of IL 6 and TNF-*α* in PRAD cells by overexpressed ARRB2. ^∗^*P* < 0.05.

## Data Availability

The datasets used and/or analyzed during the current study are available from the corresponding author on reasonable request.
